# A Neural Network Model of Smart Aging Combining Family Structure Change Factors

**DOI:** 10.1155/2022/6726475

**Published:** 2022-05-28

**Authors:** Yin-shi Jin

**Affiliations:** College of Politics and Law, Changchun Normal University, Changchun, China

## Abstract

In this paper, we analyze the changes in family structure and explore the changes in detail, based on which we construct a neural network model of smart aging. Based on the gender perspective, the individual growth model in the multilayer linear model is used to examine the effects of family structure changes on the elderly in terms of economic exchange, daily care, and emotional support. The results show that there is no significant gender difference in the family structure changes on the elderly in terms of economic exchange and daily care, but there is a significant gender difference in terms of emotional support. To solve the problem of data imbalance in the daily activity categories of the elderly, this paper resamples the data and uses different neural network models for activity recognition of the sensor data generated from the daily activities of the elderly. In this paper, the daily behavior patterns of the elderly over a while are studied by correlating three conditions of time distance, optimal path, and sensor distance to discover the daily behavior patterns of the elderly, while the abnormal behavior patterns can be well separated by EM clustering algorithm. The daily behavior of the elderly is a coarse-grained representation of their daily activities. It is not limited to a specific activity and does not require the sensor ID, trigger time, and location triggered by the activity to be consistent, but in long-term daily activity data, it abstracts the general behavior rules of the elderly activities. Through the research of this paper, the existing system is improved, and the multifaceted needs of the elderly are fully considered, from housing needs to spiritual needs, to face the current elderly care problems with a positive attitude, create a good social elderly care environment for the elderly, and realize the real elderly care.

## 1. Introduction

Modern social security theory believes that the main responsibility of old-age care should be shared by the government and families, but for a long time, the government plays a limited role in old-age care, and families are the main responsible body for the supply of old-age care resources. However, after the reform and opening up, the dramatic social transformation has affected the family structure, which has a certain impact on the family pension. Generally speaking, the structural changes of the family are mainly in terms of size, type, model, and intergenerational relationship [1]. The traditional extended family is rapidly disappearing, the family size is shrinking, and the family structure is further simplified. The phenomenon of family aging is intensifying, and the number of purely elderly families is increasing. Living patterns have changed, with the solitary model and the multigenerational model becoming the two main types of current living arrangements for the elderly. Nontraditional types of families are emerging in large numbers, such as purely elderly families, empty-nest families, intergenerational families, butch families, older single families, and single-parent families. Intergenerational relationships have changed, with the traditional patriarchal system gradually becoming equalized and intergenerational skewing common [2, 3]. In this stage of rapid development of the Internet of Things and smart hardware, we are stepping into the era of the Internet of everything [4]. The elderly care industry is a comprehensive industrial system covering the primary, secondary, and tertiary industries. It is oriented to the elderly at home, communities, and elderly care institutions and provides material and spiritual support for the elderly based on their medical, nursing, health, and nursing needs. Smart senior care systems can monitor the daily life of the elderly and give them intelligent help to solve some of the difficulties that the elderly encounter in their daily life [5].

Since many subjects are providing smart senior care services with multiple connections, they are also influenced by the internal and external environment such as policy, technology, and human environment. Therefore, this paper introduces the information ecology theory into the evaluation of the quality of information service of smart senior care, establishes the initial evaluation index of the quality of information service of smart senior care from the perspective of information ecology, and forms the formal evaluation index through verification. The questionnaire survey method is then used to empirically study the quality of information service of wisdom pensions and identify the category attributes of each index and the priority order of development to verify its rationality and validity [4, 6]. This study extends the research perspective of information ecology in the field of wisdom pension and at the same time has practical guidance significance for the improvement of information service capability of wisdom pension [7]. From a practical point of view, firstly, taking the quality of intelligent elderly care information service as the core issue, establish service quality evaluation indicators, and put forward strategic suggestions to improve the quality of intelligent elderly care information service. From the perspective of the microlevel of family structure, this paper studies its impact on rural family pension and well-being based on the change types of different family structures. Using the data of the Six-Phase Tracking Survey on Welfare Status of the Elderly, the individual growth model is used to analyze the family structure. The status quo of change and its dynamic impact on family pension and the well-being of the elderly are different from a large number of qualitative studies on this issue [8].

In this paper, we will take the family structure change factor as the research base, based on the inevitable analysis of the four subjects of government, for-profit organizations, nonprofit organizations, and the elderly in the current wisdom-based elderly care, and the daily behavior pattern of the elderly is a coarse-grained representation of their daily activities, which is not limited to a specific activity and does not require the sensor ID of the activity trigger, the time of the trigger, or the location to be consistent, but instead, it abstracts the general behavioral pattern of the elderly activities from the long-term daily activity data [9]. Finally, the different behavior patterns are classified by an EM clustering algorithm to discover different behavior patterns. The first chapter is the introduction. It mainly introduces the research background and significance of the thesis, followed by is the main research content of the thesis. The second chapter is related research, through the analysis of the current situation of domestic and foreign research, and points out the theoretical basis of this neural network model of smart aging based on family structure change factors. Chapter 3 specifically researches the neural network model of smart aging based on family structure change factors, designs the total distance calculation formula by combining the area location information of sensors, calculates the daily activity data generated by the elderly for some time, and outputs the behavior pattern of the elderly. Based on the discovered behavior patterns, the distance calculation is performed on the current activity data of the elderly to identify their abnormal behavior patterns. The principles and ideas of evaluation index construction are clarified, the framework of evaluation index of information service quality of smart elderly is designed from the perspective of information ecology, and the initial evaluation index is constructed by combining literature research and other methods. Chapter 4 is the result analysis. The results of empirical research are analyzed, and suggestions are made in combination with the four dimensions of information service ontology, information people, and information technology and information environment for constructing the evaluation index of information service quality of wisdom pension to improve the quality of information service of wisdom pension. Chapter 5 is the conclusion. It summarizes the main research contents of this paper, analyzes the shortcomings of the article, determines the focus of the subsequent research, and puts forward a reasonable outlook.

## 2. Related Research

The vast majority of domestic and foreign scholars believe that with the advancement of urbanization and the rapid transformation of the social economy, the traditional family pension function is gradually weakening, the responsibility for child support has shrunk, and the traditional family pension model will also face huge challenges [10, 11]. Kekez et al. believe that the continuation and maintenance of stem families and joint families benefit from the intergenerational interdependence in material and spirit and the balance and reciprocity of intergenerational relationships. In the long run, however, the process of modernization will eventually weaken the exchange of life care and economic and emotional exchanges between parents and children [12]. Ahmed et al. pointed out that in the context of rapid social and economic transformation, population mobility in a macro perspective is the geographical division of family members in a microenvironment, which changes the family structure. Although the economic exchanges between family members will not be interrupted, the intergenerational life care relationship will inevitably be affected by geographical restrictions [13]. Subramanian et al. identify patterns in sensor data based on activity discovery algorithms that can divide undefined classes and provide insights about behavioral patterns while learning these discovered patterns as additional classes also improves online activity recognition algorithms accuracy [14]. The advantage of using this smart pension scheme is that the elderly and patients can live comfortably at home and improve their quality of life. Smart elderly care services are mainly reflected in two points: one is to optimize the living environment and improve the quality of life of the elderly; the other is to help relieve the pressure of social public medical care [15].

Industrial upgrading and transformation, applying smart technologies to smart elderly care services, and the construction of smart elderly care are inseparable from the efforts of all walks of life. It is necessary to deploy and construct from the smart city circle, service circle, and user circle. It is recommended that relevant government departments' supervision has also been strengthened to enrich and improve various smart pension evaluation management mechanisms [16]. Jiang et al. used intelligent technology to design a comprehensive pension model for the elderly at home, which can provide basic services such as medical health and daily life to meet the daily needs of the elderly [6]. To solve the daily life problems of the elderly living alone, Nasrullah et al. integrated technologies such as medical information and home automation and designed a smart old-age care model for the elderly living alone [17]. Laadjal et al. designed a sensing system and a smart medical service model for the health monitoring problem of the elderly, which can continuously monitor their health status and provide emergency support when they need it and use feature extraction engineering to extract features such as mean, variance, entropy, correlation coefficient, and Fourier coefficient. However, some manually extracted features lack some empirical knowledge, which may lead to poor performance of the final model [18]. Therefore, in the later stage, related deep learning-based methods have been developed to automatically learn features for activity recognition, activity pattern discovery, and behavior anomaly detection [19, 20].

Through the research summary of domestic and foreign literature, the following three problems still exist in the current research on smart aging. First, most of the studies start from the macro level, lacking holistic and global thinking about the smart aging model. Secondly, the research is more concerned with the service issues of the smart senior care model. Although most scholars have found that the smart senior care model has problems such as difficulty in-service promotion, low recognition by the elderly, inability to match the quantity and quality of smart senior care service supply, and prominent contradiction between supply and demand, they have neglected the root cause of this phenomenon [21]. Third, although some scholars have recognized that the government is the main driving force in the construction of the smart senior care model and believe that the government's focus in system operation is located at the end of the overall system operation, they have ignored the drawbacks within the government itself or the interest games and political expectations among various levels of government, which have hindered the development of the smart senior care model [22]. The smart elderly care community has the unparalleled advantages of institutional elderly care and family elderly care. It can provide close-range, point-to-point elderly care services for the elderly and has been respected by many cities. However, the smart elderly care community involves multiple stakeholders, the interests of each subject are complex, and the goals are not unified, which hinders the development of the smart elderly care community. Therefore, exploring the behavioral game of multiple subjects within the smart elderly care community can better coordinate the interests of all parties, effectively promote the construction of the smart elderly care community, and provide high-quality elderly care services for the elderly. This study studies the intelligent aging neural network model based on the changing factors of family structure.

### 2.1. Performance of Family Structural Change Factors

Smaller families enhance the elderly's sense of self-reliance and ability to live independently. Changes in social thinking and culture and the popularity of new social lifestyles have not only changed the mindset of young people in the region but also of the elderly, who have gradually accepted the small family style of living, have changed their expectations of their children's retirement, and have begun to actively plan for their savings in old age. Smaller families have a direct impact on reducing intergenerational and peer conflicts in families. Since living separately from their children avoids certain family disputes, they can better maintain family intimacy. According to psychology, the relationship between people is directly related to the distance between them, and too much interaction may intensify conflicts over family matters, which is not conducive to the maintenance of good intergenerational relationships. Changes in family structure have improved the common mother-in-law-daughter-in-law conflict to some extent. Traditionally, mother-in-law-daughter-in-law conflicts were frequent in extended family relationships, but in the current situation where a large number of young and strong male laborers go out to work, daughters-in-law have taken on the burden of caring for their in-laws and have achieved understanding and tolerance in supporting each other. In terms of the environment for the elderly to age, a stable and calm environment is more conducive to the physical and mental health of the elderly. Small families are more suitable for the physiological and psychological rhythm of the elderly than traditional large and noisy families [23, 24].

The number of older adults living alone due to widowhood is slightly higher for men than for women. The change of second- and third-generation direct line families to single-person households was mainly due to the separation of the elderly from their children for work-related reasons. The reasons for the change from direct intergenerational households to single-person households are various, including the growing age of the elderly and the removal of grandchildren by their out-of-town children. It should be noted that the change from direct intergenerational households to single-person households is mainly due to the female elderly. In conclusion, the proportion of single-person households in all family structure types is on the rise, mainly because the splitting of the couple's nuclear family has increased the proportion of single-person households, followed by the change from direct two-generation families, direct three-generation families, and direct intergenerational families to single-person households, which has led to the increasing proportion of single-person households [25]. The behavioral characteristics of the elderly have a very important impact on the interaction design of subsequent mobile devices, which will help the subsequent design research work. The direct and indirect factors influencing the behavior of the elderly are analyzed in Table 1.

Aging scenarios need to be analyzed in conjunction with the types of aging, taking the three existing types of aging: home aging, community aging, and institutional aging. Senior care institutions generally provide more services tailored to the needs of the elderly, but there are still elderly people who need to live at home to age in place. Aging at home is closer to the deep-rooted ideas of the people, respecting both the inherent concept of family life and being accepted by more elderly people and families. Home aging and community aging will produce crossover, and the author has made a scene classification for this part of the elderly aging scene (Figure 1) and will do user research on the natural scene in the aging scene below. According to the classification of user experience field scenarios, in-depth analysis is carried out against pension scenarios. Based on the anthropological characteristics of the elderly group, the interactive behavior of the elderly is deeply studied, and the direct and indirect factors affecting the interactive behavior of the elderly are summarized. Changes in family structure will affect the family pension and the well-being of the elderly.

### 2.2. Construction of Neural Network Model for Smart Aging

In this paper, the daily behavior patterns of users are discovered based on processing and analyzing the unlabeled sensor data collected in smart homes. In this paper, the daily behavior patterns of users are modeled by combining temporal information with sensor information using a dynamic time regularization algorithm and multiple associated restrictive conditions. Firstly, a sequence is initialized for the daily behavior pattern of the elderly, as shown in (1), where *Q*(*x*) represents a behavior pattern. *Q*(*x*) is composed of a sequence of hidden activities of the elderly's daily activities, i.e., it consists of multiple sensor event sequences. In this paper, we use the designed distance calculation method to calculate the daily two-two corresponding time distance and sensor distance in the experimental data and then use the EM clustering algorithm to cluster the fusion of the two distances, and the similar behavioral patterns are clustered into one behavioral pattern.

(1) $$\begin{array}{c} Q\left(x\right)=\left\{\zeta_{1}^{Q\left(1\right)},\zeta_{2}^{Q\left(2\right)},\cdots ,\zeta_{N}^{Q\left(N\right)}\right\}. \end{array}$$

The data generated by the sensor is divided into two parts for the study, which include time distance and sensor distance. The temporal distance and sensor distance are calculated using a custom distance formula. The total distance is the fusion of the two sums, i.e., the smaller the distance, the more likely it is that the daily behavior pattern belongs to a behavior pattern. As shown in (2), *D*(*S*(*D*_*i*_, *D*_*j*_)) is the total distance between day *i* and day *j* integrated by temporal distance and sensor distance, *D*(*T*(*D*_*i*_, *D*_*j*_)) is the temporal distance between day *i* and day *j*, *Q*(*D*_*i*_)+*Q*(*D*_*j*_) is the total number of sensor events occurring on the day *i* and day *j*, and *D*(*E*(*Q*(*D*_*i*_)) is the sensor distance between day *i* and day *j*.

(2) $$\begin{array}{c} D\left(S\left(D_{i},D_{j}\right)\right)=D\left(T\left(D_{i},D_{j}\right)\right)+\frac{D\left(E\left(Q\left(D_{i}\right)\right.\right)}{Q\left(D_{i}\right)+Q\left(D_{j}\right)}. \end{array}$$

Simplifying the notation gives (3), in which *D*_*i*_ represents day *i* and *D*_*j*_ represents day *j*.

(3) $$\begin{array}{c} H\left(D_{i},D_{j}\right)=D\left(T\left(D_{i},D_{j}\right)\right)+\frac{D\left(E\left(Q\left(D_{i}\right)\right.\right)}{Q\left(D_{i}\right)+Q\left(D_{j}\right)}. \end{array}$$

A neural network is processed on all the data to analyze the relationship between the temporal information of the behavioral data. After processing, the temporal distance is calculated for any two days by (4).

(4) $$\begin{array}{c} H\left(T\left(D_{i},D_{j}\right)\right)=\text{DWT}\left(T\left(D_{i},D_{j}\right)\right)+\sum_{m=1}^{N}\text{DWT}\left(D\left(m\right)\right). \end{array}$$

The distance between the first data of any two days is shown in (5). Based on the sensor data collected in the smart home environment, the daily activities of the elderly are identified and studied based on the deep learning model. In order to solve the problem of unbalanced data of the elderly's daily activity categories, the data are resampled, and different neural network models are used to identify the sensor data generated by the elderly's daily activities.

(5) $$\begin{array}{c} H\left(T\left(D_{i},D_{j}\right)\right)=\left\|\frac{\sqrt{T\left(D_{i},D_{j}\right)+T\left(D_{j},D_{i}\right)}}{2}\right\|. \end{array}$$

There are many paths from the first node to the last node, which are defined as H paths, each of which is a regular path for *D*_*i*_ and *D*_*j*_ days, and what we want to do in this paper is to find the least costly path from H paths as the optimal path corresponding to the shortest distance, where K is the number of path nodes taken by the regularized path, *N*(*D*_*i*_) represents the total number of sensor events in *D*_*i*_ days, *N*(*D*_*j*_) represents the total number of sensor events in *D*_*j*_ days, *P*(*i*) is one of the regularized paths, and N represents the optimal path after regularization.

(6) $$\begin{array}{c} \left\{\begin{array}{c} Q=\sum_{i=1}^{N}Q\left(i\right)+\beta {}^{*}p,\\ \begin{array}{c} MIN\left(N\left(D_{i},D_{j}\right)\right)\leq N\leq N\left(D_{i}\right)+N\left(D_{j}\right)\\ 1\leq p\leq H \end{array}. \end{array}\right. \end{array}$$

For the elderly, it is assumed that when the elderly “choose” to join the strategy, the return is *A*(1); when they take the “no-choice” strategy, the return is *A*(2); and the average return is $\overset{⟶}{A}$. Then, the elderly “choose,” the expected return *A*(1) when the elderly “opt-in,” the expected return *A*(2) when they “opt-out,” and the average return *p* are shown in (7). In the case that the government chooses to strictly regulate and the for-profit organizations choose to operate passively, even if the government gives subsidies to the elderly to participate, the spiritual benefits that the elderly reap from the services in the for-profit organizations are still less than the costs they pay, and the optimal strategy is when the elderly choose not to choose the services in the smart retirement community.

(7) $$\begin{array}{c} \left\{\begin{array}{c} A\left(1\right)=F\left(W\left(3\right)-W\left(1\right)-W\left(4\right)+W\left(2\right)\right)+\frac{\alpha {}^{*}W\left(\beta \right)+W\left(4\right)-W\left(2\right)}{3},\\ \begin{array}{c} A\left(2\right)=\sqrt{\sum_{i=1}^{4}W{\left(i\right)}^{2}},\\ \overset{⟶}{A}=\xi A\left(1\right)+\left(1-\xi \right)A\left(2\right). \end{array} \end{array}\right. \end{array}$$

For the government, let the government's return when adopting the “strict regulation” strategy be *B*(1) and the return when adopting the “lax regulation” strategy be *B*(2). The average return is $\overset{⟶}{B}$. Then, the government's return from adopting the “strict regulation” and “lax regulation” strategies, as well as the average return, are shown in (8). When the government chooses to strictly regulate, the government's reputation gain and penalty gain are greater than the government's cost in strictly managing the evaluation of smart senior care, and the government chooses “strict regulation” as the optimal strategy.

(8) $$\begin{array}{c} \left\{\begin{array}{c} B\left(1\right)=X\left(3\right)-X\left(R\right)-X\left(C\right)+X\left(2\right)+\frac{Y\left(S\left(X\right)+S\left(C\right)+S\left(R\right)\right)}{2}-\mu {}^{*}W\left(X\right),\\ \begin{array}{c} B\left(2\right)=\sqrt{\sum_{i=1}^{4}X{\left(i\right)}^{2}+W{\left(i\right)}^{2}},\\ \overset{⟶}{B}=\psi B\left(1\right)+\left(1-\psi \right)B\left(2\right). \end{array} \end{array}\right. \end{array}$$

When a profit-making organization operates, the return is *C*(1) when it adopts a “positive management” strategy, and the average return is *C*(2) when it adopts a “negative management” strategy, then the profit-making organization chooses “positive management”, and the expected returns and the average returns of the profit organization choosing “active” and “negative” operation are shown in (9). When the profit of the profit-making organization in negative operation is greater than the profit of the profit-making organization in positive operation, and the cost of government penalties is still less than the profit of the profit-making organization in negative operation when the government strictly regulates the profit-making organization, then the profit-making organization is the optimal strategy when it chooses negative operation.

(9) $$\begin{array}{c} \left\{\begin{array}{c} C\left(1\right)=Z\left(2\right)-Z\left(H\right)-Z\left(Q\right)+\frac{H\left(Q\left(Z\right)+Z\left(2\right)+Q\left(U\right)\right)}{3}-\varpi {}^{*}Z\left(1\right),\\ \begin{array}{c} C\left(2\right)=\sqrt{\sum_{i=1}^{4}Z{\left(i\right)}^{2}+Y{\left(i\right)}^{2}},\\ \overset{⟶}{C}=\rho C\left(1\right)+\left(1-\rho \right)C\left(2\right). \end{array} \end{array}\right. \end{array}$$

The model examines the differences in the development trend of the elderly's life satisfaction among individuals. Since this paper assumes that the elderly's life satisfaction changes nonlinearly with age, the interaction terms of age, age square, and age and family structure changes are included in the model, and time-varying variables (individual characteristics of the elderly and intergenerational support) are included in the model.

### 2.3. Evaluation of the Quality of Smart Aging

The information service quality evaluation is the evaluation of both service subjects and service users, and the information service subjects and information service users are the first-level indicators under the information technology dimension; the information service platform and intelligent products derived from information technology are the centralized manifestations of the wisdom of senior care service [26]. The information service platform and intelligent products derived from information technology are the centralized manifestations of the wisdom of senior care service, and two-level indicators are set up under the information technology dimension, namely, technology platform and technology products; the environment in which the wisdom senior care information service is located include two-level indicators, namely, the internal environment close to the information person and the external environment far from the information person.  Table 2 shows the evaluation indexes of the quality of the information service of the smart elderly.

In combination with the practical application of hierarchical analysis, it is possible to identify the weights of the indicators at different levels and to calculate the evaluation results. The specific implementation steps of the hierarchical analysis method have been outlined in detail in the previous paper, i.e., constructing a multilevel indicator system, combining expert opinions and literature data, selecting the corresponding elements in the hierarchical elements for comparison, thus constituting a judgment matrix, and finally solving for the ranking weights. During the field visits of the wisdom pension system wisdom pension evaluation, it was found that the implementation of the corresponding wisdom pension evaluation management system was unsatisfactory due to the poor evaluation awareness of the project wisdom pension evaluation managers. A personal growth model was established in the multilevel linear model to investigate the impact of changes in family structure on the health self-assessment of the elderly; Secondly, the development trend of life satisfaction and family structure of the elderly are investigated by establishing a multilayer linear model in the personal growth model.

In the process of implementation, the quality evaluation of smart senior care needs to be measured, collected, organized, and analyzed with the help of the quality evaluation questionnaire, the quality evaluation table of smart senior care (Table 3), and the quality evaluation result in analysis table of smart senior care, which aims at classifying the attributes of the investigated quality indicators and suggesting strategies to improve the service quality according to the classification results.

## 3. Analysis of Results

### 3.1. Analysis of the Neural Network Model of Intelligent Aging

By accessing the historical data of node detection at the platform side, it can be seen that the real values of node Temp value and Humi value collection results generated by the exported Excel table are compared with the algorithm model for training test to obtain the model prediction internal implicit state of the node. The comparison results between its real value and the prediction results of the smart aging neural network model are shown in Figure 2, where the horizontal axis indicates the test time, the vertical axis indicates the node state, “1” indicates the abnormal error state, “3” indicates the normal state, and “5” indicates the state of drastic parameter changes. By comparing the real value of node detection with the predicted result of the node state of the smart aging neural network model, the future changes of the sampled data of the system can be effectively predicted. According to the model analysis, when the measured application scenario has significant parameter changes in the future moments, to improve the accuracy of the system application to maintain the system power consumption stability, increase the overall data collection time so that the system can effectively complete the parameter monitoring in real time.

The time distance between the first day and the remaining days is calculated based on the time distance as shown in Figure 3, where Figure 3(a) represents the time distance information of the elderly in one month, the horizontal axis represents the plotted attribute distance, and the vertical axis represents the range of distance values. It can be seen that there are three outlier points in the figure, which coincide with the previously plotted data, and these three days are anomalous data with an average value of around 400. Based on the information shown in Figure 3(a), we can obtain the three points in red in Figure 3(b) as outliers, and Figure 3(b) represents the line graph of the time distance between D1 and the rest of the days. The value of the horizontal axis indicates the information on the number of days; the vertical axis indicates the value of the distance between D1 and the rest of the days.

The activities of Leave_Home and Enter_Home are correlated, so in this paper, the activity times of Leave_Home and Enter_Home are combined and plotted as shown in Figure 4, where the left graph of Figure 4 uses the start time of Leave_Home as the *X*-axis and the start time of Enter_Home as the Y-axis, and the right graph of Figure 4 uses the start time of Enter_Home as the *X*-axis and the time difference between the start time of Enter_Home and Leave_Home as the *Y*-axis. From the graph, we can see that the elderly people all leave home after 9:00 am and return home around 9:00 pm. The longer time range of leaving home is between 9:00 and 12:00.

The family-oriented home care method is still the main form of old-age care, and the government-oriented social old-age security method can only be used as a supplementary means of family old-age care but not as a substitute for family old-age care. First of all, the coverage and amount of social pension guarantee are very limited and far from meeting the needs of the elderly in the region. Secondly, family pension is still the effective pension method in the region, and the family pension is irreplaceable in terms of blood kinship culture, as shown by the fact that most of the elderly are still willing to live with their children and rely on them for their pension. Finally, after entering the aging society, with limited public resources, the state's support for regional old-age care can be in the form of auxiliary family support in addition to basic old-age security pension. Especially in the period of social transition, the unevenness of social and economic development makes family pensions exist in an unstable state, but this does not mean the demise of family pensions. This phase of building the pension system should be an expansion and supplement to the existing system rather than suppression and replacement.

### 3.2. Evaluation Analysis of the Quality of Intelligent Aging

Regression results for the effect of family structure change on older adults' access to financial support are presented in Figure 5. In single person families, couples' nuclear families, and direct intergenerational families, elderly fathers receive a higher level of economic support from their children, while for elderly fathers and mothers, when the family changes to direct intergenerational families, elderly fathers and mothers receive the most economic support. In the benchmark period, the elderly whose family structure belongs to intergenerational lineal families, whether elderly fathers or elderly mothers, can receive financial support. The initial mean value of the level of financial support was higher for both elderly fathers and mothers. Older adults received lower levels of financial support compared to younger older adults; those who were married received higher levels of financial support than those who were not, especially older fathers; older fathers with independent financial income received less financial support than those without independent financial income; older adults with more children also received higher levels of financial support, and the more daughters there were, the more financial support older mothers received. Educated older fathers received higher levels of financial support than uneducated older fathers; however, the effect was not significant for older mothers; older fathers who worked in agriculture received higher levels of financial support, while older mothers who worked in agriculture received less financial support.

The effect of changes in family structure on the life satisfaction of the elderly is a gradual accumulation process. Although changes in family structure are positively correlated with life satisfaction, however, the negative effect of changes in family structure on the life satisfaction of the elderly is gradually accentuated as the elderly grow older. Based on the regression results of the quality evaluation of smart aging, the effects of changes in different family structures on life satisfaction were predicted as shown in Figure 6. Figure 6 shows that the life satisfaction of the elderly changes nonlinearly with age, and there is a significant difference in the life satisfaction of the elderly under the change of different family structures in the lower age stage, and this difference gradually decreases with age. This may be because when the family structure changes to a single-person household, the problem of lack of elderly resources becomes more prominent, especially the possibility of increasing loneliness and depression, and thus, the life satisfaction is lower and decreases faster with age.

When nonprofit organizations adopt the joining strategy, the more the nonprofit organizations gain from it, the more the nonprofit organizations' enthusiasm to join the for-profit organizations will increase; at this time, the H1 parameters are set to 10 and 12, as shown in Figure 7. Similarly, the enthusiasm of for-profit organizations to improve senior care services also increases, which plays a positive role in the service improvement of for-profit organizations. At the same time, the profitability of for-profit organizations will increase as the service improvement increases, which will lead to a win-win situation for both nonprofit organizations and for-profit organizations as shown in Figure 7. Figure 7 is a change trend chart, and we can see the growth trend. With the continuous increase in the investment and supervision of nonprofit organizations, in order to avoid punishment, the enthusiasm of for-profit organizations to improve services is also increasing.

When the family structure changed to single family, couple nuclear family, and intergenerational straight family, there was a positive correlation with the self-evaluation of the elderly's health, and when the family structure changed to a second-generation straight family, it was positively related to the self-evaluation of the elderly's health but not significant. There was a significant positive correlation with the elderly's health self-assessment when it was a three-generation straight family. In terms of life satisfaction, the negative impact of changes in family structure on the life satisfaction of the elderly is gradually prominent. Although changes in family structure are positively correlated with the life satisfaction of the elderly, as the elderly grow older, it is positive. The correlation gradually weakened and had a negative impact. With the increase of age, no matter what kind of family changes, the life satisfaction of the elderly decreases nonlinearly, and the difference of the influence of different family structure changes on the life satisfaction of the elderly gradually decreases with the increase of age.

## 4. Conclusion

Changes in the family structure were positively correlated with older adults' health self-assessment when the family structure changed to a single-person family, a couple's nuclear family, and an intergenerational direct family; when the family structure changed to a two-generation direct family, it was positive but not significantly correlated with older adults' health self-assessment, and when the family structure changed to a three-generation direct family, it was significantly and positively correlated with older adults' health self-assessment. In terms of life satisfaction, the negative effect of changes in family structure on the life satisfaction of older adults was gradual. Although changes in family structure were positively correlated with the life satisfaction of older adults, the positive relationship diminished and became negative as older adults aged. The difference between the changes in family structure and the life satisfaction of the elderly decreases gradually with age. The evaluation methods are different but have the same purpose, i.e., to identify the evaluation indexes that need to be developed in a priority manner. Although the indicators are not weighted in this paper, they can be incorporated into the research process in future studies as the smart senior care information service continues to mature. In the simulation analysis, easier protocols can be chosen to realize the connection between terminal devices and the platform, increasing the processing of data by the platform, making the monitoring application of data richer, while the platform connects other clients with the help of the current big data analysis technology.

## Figures and Tables

**Figure 1:** Classification of elderly care scenarios.

**Figure 2:** Comparison of model prediction results and true values.

**Figure 3:** Distance information.

**Figure 4:** Presentation of time information for leaving home and returning home activities.

**Figure 5:** Estimates of multilayer linear models of the impact of changes in family structure on family retirement based on gender differences.

**Figure 6:** Evaluation results of life satisfaction of the elderly under the change of family structure.

**Figure 7:** Simulation analysis results under the influence of different input parameters.

**Table 1:** Influencing factors.

Influencing factor number	Family structure features	Direct influence factors	Indirect influence factors
1	Instability	Interactive scene change	Reduced adaptiveness of perception systems
2	Objective scenario influence		Vision, hearing, memory loss
3			
4	Successful completion of the act	Interaction time limit	Neurotransmitter degeneration
5			Response time is prolonged

**Table 2:** Evaluation indexes of information service quality of wise senior citizens.

Evaluation number	Evaluation dimension	First-level evaluation index	Second-level evaluation index
1	Information service ontology	Information characteristics	B1
2		Service features	B2
3	Information person	Information service subject	B3
4		Information service users	B4
5	Information technology	Technology platform	B5
6		Technical products	B6
7	Information environment	Internal environment	B7
8		External environment	B8

**Table 3:** Smart aging quality evaluation table.

Quality rating options		Negative question				
		Very satisfied	Satisfy	It does not matter	Reluctantly accepted	Dissatisfied
Positive question	Very satisfied	A	A	F	C	D
	Satisfy	B	D			
	It does not matter	C	B	E	E	D
	Reluctantly accepted	C	E	F	A	F
	Dissatisfied	A	C	C	B	A

A: required quality, B: expected quality, C: charm quality, D: irrelevant quality, E: reverse mass, F: suspicious result.

## Data Availability

The data used to support the findings of this study are available from the corresponding author upon request.
